# MicroRNA miR-147b promotes tumor growth via targeting UBE2N in hepatocellular carcinoma

**DOI:** 10.18632/oncotarget.23120

**Published:** 2017-12-09

**Authors:** En Zhang, Qin Liu, Yong Wang, Hui Wang, Li He, Xiuli Jin, Ning Li

**Affiliations:** ^1^ Department of Gastroenterology, The Second Affiliated Hospital of Shenyang Medical College, Shenyang 110035, China; ^2^ Department of Gynecology and Obstetrics, Seventh People's Hospital of Shanghai University of TCM, Shanghai 200137, China; ^3^ Department of Infectious Diseases, Huashan Hospital, Fudan University, Shanghai 200040, China

**Keywords:** hepatocellular carcinoma, tumor growth, ubiquitin-conjugating enzyme E2N (UBE2N), miR-147b, microRNA

## Abstract

As the subfamily of noncoding RNA, microRNAs (miRNAs) broadly regulate the development of cancers, while their dysregulation and function in human hepatocellular carcinoma (HCC) remains largely unclear. Here, we found the expression level of microRNA-147b (miR-147b) is increased aberrantly in HCC tumor tissues, and its expression positively correlates to the tumor severity. In both MTT and colony formation assay, knockdown of miR-147b dramatically inhibits *in vitro* proliferation of HCC cell lines. More interestingly, we also performed *in vivo* tumorigenesis assay and found that miR-147b can regulate *in vivo* tumorigenesis in nude mice xenograft models. The ubiquitin-conjugating enzyme E2N (UBE2N) was identified directly and functionally targeted by miR-147b. The mRNA level of UBE2N is increased in HCC tumors or cell lines. Restoring UBE2N expression level in tumor cells leads to inhibition of cell proliferation, which mimics the effect upon miR-147b knockdown in the same cells. These data elucidated the oncogenic role of miR-147b in HCC development and progression with therapeutic target potentials.

## INTRODUCTION

Hepatocellular carcinoma (HCC) is one kind of primary liver cancers with high mortality, it is the most common type of cancer worldwide, especially in Asia, African and south Europe [1]. Although some risk factors for HCC have been identified, such as hepatitis B or C viruses infection, overdrinking of alcohol et al are all involved in HCC, however, the main part of molecular mechanisms underlying HCC development remain poorly understood, which drawbacks the development of novel therapeutic approaches. Therefore, the elucidation of the molecular pathways involved in HCC will help the development of new therapeutic options [2–4]. Although many protein-coding genes have been reported to involve in the pathogenesis of HCC, the critical role of microRNA (miRNA), still kept largely undefined.

MicroRNAs belong to the family of noncoding RNAs, it is encoded by cell genome with 22 nucleotides in length, miRNA can posttranscriptional regulate gene expression both in plants and animals. It represses gene expression by degrading mRNA or terminating translation. Since the seed sequence of one miRNA can base paired with multiple different mRNA molecules, this characteristics enable the miRNA family members can regulate even up to one third of the protein coding transcripts in the whole human genome. So it attracted broad attention and interests of the researchers to uncover their functions in biological process and all kinds of disease conditions. A number of studies have demonstrated that miRNAs have been dysregulated and functionally involved in carcinogenesis [5]. In HCC, previous reports also found the upregulation or downregulation of miRNA, which indicated that their functions were also as important as the protein coding genes [6].

Both the expression and the function of MiR-147b is poorly studied, only one recently report found that by targeting ADAM15, miR147b is involved in endothelial barrier function [7]. However, its function in tumorigenesis remains totally obscure. Here we report that the aberrantly upregulation of miR-147b in HCC tumor samples, further functional study demonstrates miR-147b promote HCC tumor growth by targeting ubiquitin-conjugating enzyme E2N (UBE2N).

## RESULTS

### Up-regulation of miR-147b was found in HCC tumor samples and cell lines

First of all, we checked the expression of miR-147b in HCC tumor samples, relative adjacent liver samples, and nontumor controls. Results from northern blot analysis show an enhanced quantity of miR-147b in HCC group, compared to those in adjacent tissues and nontumor controls (Figure 1A). Statistical analysis of the band density shows the significant up-regulation of miR-147b in HCC group (Figure 1B). Quantitative PCR (qPCR) analysis reveals that miR-147b showed a 2-fold upregulation in the HCC group compared to nontumor controls or HCC adjacent tissues (Figure 1C). To further explore if miR-147b is involved in HCC pathogenesis, the expression level of miR-147b was analyzed in HCC tumor samples with different AJCC disease stages [8, 9]. The results showed a 2-fold and 3-fold increase in T1- and T2-stage, and a 4-fold upregulation in T3-stage compared to control sample (Figure 1D). Moreover, we also compared miR-147b expression levels with HCC tumor volumes and found that the larger the tumor volumes, the higher expression of miR-147b existed, which demonstrated miR-147b closely correlates with tumor volumes (Figure 1E). Compared to L02, the normal liver cells, the expression level of miR-147b in HepG2 and Huh 7 was also found significantly increased (Figure 1F). The above results demonstrate that miR-147b is up-regulated in HCC tumors, its expression is positively correlated to disease severity.

**Figure 1:** Up-regulation of miR-147b was found in HCC tumor samples and cell lines **(A, B)** Northern blot detection of miR-147b in nontumor control, adjacent tissues and HCC tumor tissues, the representative pictures (A) and statistics data (B) were shown. **(C)** qPCR detection of miR-147b level in different type of tissues. **(D-E)** qPCR detection of miR-147b expression level in HCC tissues in different disease stage (D) or with different tumor volume (E). **(F)** qPCR detection of miR-147b level in liver cell lines. snRNA U6 expression used as the loading control. ^*^P<0.05, ^**^P<0.01, ^***^P<0.001.

### Knockdown of miR-147b inhibits *in vitro* HCC tumor cell proliferation

As demonstrated above, miR-147b is significantly upregulated in HCC tumors and cell lines, we further wonder if miR-147b play critical role in regulate HCC tumorigenesis. After transfected with antisense oligo (anti-miR-147b), HepG2 and Huh 7 showed significantly decreased expression of miR-147b (Figure 2A), and cell proliferation was analyzed, results from MTS assay indicated significantly inhibited cell proliferation of both HepG2 (Figure 2B) and Huh 7 (Figure 2C) upon the knockdown of miR-147b. Cell proliferation was further detected by colony formation, and in both HepG2 and Huh 7, colony numbers were greatly reduced when miR-147b was knockdown (Figure 2D and 2E), these data showed that miR-147b plays a critical role in promoting HCC tumor cell lines proliferation.

**Figure 2:** Knockdown of miR-147b inhibitsl proliferation in HCC tumor cells MiR-147b was knockdown in HepG2 and Huh 7 by anti-sense oligo (Control or anti-miR-147b). **(A)** mRNA level of miR-147b in HepG2 and Huh 7 after oligo transfection. **(B-C)** Proliferation of HepG2 (B) and Huh 7 (C) was measured using the MTS assay. **(D-E)** Formation of colonies in HepG2 and Huh 7 transfected with oligos, the representative pictures (D) and statistics data (E) were shown. ^***^P<0.001.

### Knockdown of miR-147b inhibits *in vivo* tumor growth in nude mice xenograft models

We further construct the nude mice xenograft models to check if miR-147b can also regulate *in vivo* tumor growth. After transfected with anti-miR-147b, miR-147b mimic, or control oligos, HepG2 and Huh 7 cells were injected into nude mice subcutaneously. MiR-147b expression level in HepG2 and Huh 7 cells after oligo transfection were verified by qPCR (Figure 3A). *in vivo* growth of HepG2 and Huh 7 cells in nude mice were detected by measuring the tumor volumes each week post-injection, we found that, compared to the control group, the tumor growth in miR-147b knockdown group (anti-miR147b) was significantly decreased, while the growth rate in miR-147b overexpression group (miR-147b mimic) was significantly enhanced (Figure 3B, 3C). Six weeks after inoculation, we found both the volume and weight of the tumor were decreased significantly in miR-147b knockdown group (anti-miR147b), and were increased significantly upon miR-147b overexpression (miR-147b mimic) (Figure 3E). All of these data demonstrated that miR-147b can also regulate *in vivo* HCC tumor growth.

**Figure 3:** Knockdown of miR-147b inhibits in vivo tumor growth After transfected with different oligos, HepG2 and Huh 7 cells were injected into nude mice subcutaneously. **(A)** qPCR detection of miR-147b and UBE2N expression levels in HepG2 and Huh 7 cells after oligo transfection. **(B, C)** Tumor growth of HepG2 (B) or Huh 7 (C) cells in nude mice. **(D, E)** At the end of experiments in B and C, the tumors were separated and the pictures of tumors were represented (D) and the tumor weight were measured and analyzed (E). ^***^P<0.001.

### UBE2N was identified as miR-147b target

To explore the underlying mechanisms of miR-147b regulation of HCC proliferation, we further investigate which target gene mediates the function of miR-147b. Several miRNA target predicting algorithm including Targetscan (targetscan.org); miRanda (microrna.org); and Pictar (mdc-berlin.de) were applied to predict for potential miR-147b targets (Figure 4A). UBE2N was predicted to have potential binding sites in its 3’-UTRs with high fidelity (Figure 4B). To verify the direct binding between the potential sites in UBE2N’s 3’-UTR and miR-147b, the 3’-UTR was cloned and inserted into the luciferase reporter vector pGL3, and then transfected these plasmids with pll3.7 vectors which overexpressed WT miR-147b or mutated miR-147b. The luciferase activities of UBE2N 3’-UTR were repressed by WT miR-147b significantly (Figure 4C). As miR-147b was upregulated in HCC tumor samples, we further tested UBE2N expression levels in HCC tumor tissues, relative adjacent tissues and normal livers. The results showed that the mRNA level of UBE2N was decreased significantly in the tumor tissues compared to that of the adjacent or health tissues (Figure 4D). We further detected UBE2N expression level in HCC tumor cells or normal L02 cell, the data showed that UBE2N was also down-regulated in both HepG2 and Huh 7, compared to the L02 cell line (Figure 4E). To demonstrate the direct regulation of UBE2N by miR-147b, we manipulated the expression level of miR-147b in both HepG2 and Huh 7 cells, and we found overexpression of miR-147b significantly decreases UBE2N protein level, while knockdown of miR-147b increases UBE2N protein level significantly in both HepG2 and Huh 7 cells (Figure 4F, 4G). Finally, we detected the protein level in HCC and adjacent controls, and the results further verified that UBE2N is decreased significantly in HCC, compared to the adjacent controls tissues (Figure 4H). These results demonstrated UBE2N as the direct functional target gene of miR-147b during HCC pathogenesis.

**Figure 4:** UBE2N was identified as miR-147b target **(A)** UBE2N gene was predicted as the potential miR-147b target predicted by several programs. **(B)** MiR-147b binding elements in the 3’-UTR of UBE2N and the mutated sites. **(C)** Luciferase reporter analysis of direct binding of miR-147b to the 3’-UTR of UBE2N. **(D-E)** mRNA expression levels of UBE2N in clinical samples (D) and HCC cell lines (E). **(F-G)** After transfected with scramble control, miR-147b mimic and anti-miR-147b oligoes, protein levels of UBE2N in HepG2 (F) and Huh 7 (G) cell lines were detected with specific antibody. **(H)** Protein level of UBE2N in adjacent tissues and HCC tumor tissues were analyzed by western blot. ^**^P<0.01, ^***^P<0.001.

### Overexpression of UBE2N suppressing HCC cell proliferation

The function of target gene in HCC tumorigenesis was further investigated. qPCR verified that these overexpression vectors efficiently overexpressed the target UBE2N in both HepG2 and Huh 7 (Figure 5A). MTS assay indicated overexpression of UBE2N significantly suppressed cell proliferation (Figure 5B, 5C). The clone formation assay further verified that the results from MTS assay (Figure 5D, 5E).

**Figure 5:** Overexpression of UBE2N suppressing proliferation of HCC tumor cells **(A)** UBE2N expression levels were detected in HepG2 and Huh 7 cells after transfected with different vectors. **(B-C)** Cell proliferations of HepG2 (B) and Huh 7 (C) were measured using the MTS assay. **(D-E)** Formation of colonies in HepG2 and Huh 7 transfection, the representative pictures (D) and statistics data (E) were shown. ^***^P<0.001.

## DISCUSSION

Both the expression profile and function of miR-147b were less-studied, recently, only one report showed that miR-147b was involved in regulating endothelial barrier function. As another member of the same cluster to miR-147b, miR-147 was reported to involved in several tumor progresses, Lee et al find that miR-147b induced MET and cell cycle arrest in both colon and lung cancer cells [10]. MiR-147 was also found decreased in NSCLC tumors and sera than those in control patients. Low serum level of miR-147 is correlated with tumor metastasis, LNM, and tumor size [11]. Zhang and colleagues reported that miR-147 inhibited breast cancer migration and proliferation by targeting the Akt/mTOR pathway [12]. Although the above data indicated that miR-147 participates in tumorigenesis, however, the role of miR-147b was largely unexplored, here we report for the first time that miR-147b was dysregulated during HCC pathogenesis and positively regulated HCC tumor cell proliferation.

MiRNA exerts function indirectly through binding to the specific elements in target genes’ 3’-UTR, then further degrade mRNA or inhibit protein translation of targets [13]. A disintegrin and metalloproteinase15 (ADAM15) was the first identified miR-147b target gene reported recently [7]. In this study, we identified that UBE2N was directly targeted by miR-147b. UBE2N is a ubiquitin-conjugating enzyme [14]. Ubiquitination process is finished by ubiquitin-activating enzymes including E1s, E2s, and E3s [15–17]. UBE2N is one E2 ubiquitin-conjugating enzyme, and critically involved in DNA post-replication repair [18]. As ubiquitinated proteins will be degradated by cells, so the inhibition of UBE2N in tumor cell will lead to tumorigenesis is reasonable [19]. And here we found that in HCC tumors and cell lines miR-147b was upregulated and targeted UBE2N, which further will lead to the downregulation of UBE2N, and our data did verify that UBE2N was really downregulated in the HCC tumors or HCC cell lines. And the negative correlation between miR-147b and UBE2N further support UBE2N act as the functional target of miR-147b.

More interestingly, the function of UBE2N in HCC tumorigenesis was undefined, and here we found that overexpression of UBE2N significantly represses HCC tumor cells proliferation both in HepG2/Huh 7 cells. This finding not only further support UBE2N act as the real target of miR-147b, but also revealed for the first time that UBE2N functionally participates in tumor suppression, at least in HCC.

In summary, we demonstrated miR-147b was upregulated in HCC tissues or cell lines. Knockdown of miR-147b repress HCC cell growth both *in vitro* and *in vivo*. The UBE2N was identified as the real target of miR-147b. And UBE2N’s role during HCC tumorigenesis was also demonstrated here. Our data indicated an oncogenic role for miR-147b in HCC development with therapeutic potentials.

## MATERIALS AND METHODS

### Cell culturing, plasmid construction, synthetic RNA oligo

HepG2, Huh 7, 293T, L02 were cultured in DMEM medium with 10% FBS (Invitrogen) under 5% CO_2_ at 37 °C.

For miR-147b over-expression, a 300 base pairs genomic region covering pre-miR-147b was amplified and ligated with the pll3.7 vector [20]. For UBE2N overexpression, its ORF region was amplified and inserted into pcDNA3 plasmid. The 3’-UTR of UBE2N was amplified and ligated with the pGL3 reporter plasmid. Mutated vectors were constructed using the Kit from Agilent.

MiR-147b mimic oligos (ATCGTCTTCGTAAA GGCGTGTG), anti-miR-147b oligos (CACACGCCTTT ACGAAGACGAT), and control oligos (AGTTCTTGCAC GGAACGTACG) were synthesized by Shanghai Gene-Pharma Co.

### Clinical tissues

Tumor or control tissues were collected from the Second Affiliated Hospital of Shenyang Medical College (Shenyang, China) according to 2002 criteria of AJCC [8]. All samples had similar proportions of sex (about 50% each) and ages (19∼66 years old). The study acquired the approval of the Research Ethics Committee of the Second Affiliated Hospital of Shenyang Medical College. All donors had signed informed consent.

### Quantitative real-time PCR (qPCR) and northern blot

Total RNA was extracted with TRIzol (Roche) following the manual. MiR-147b was quantified with TaqMan probe and qPCR from ABI with U6 as the loading control. For mRNA quantification, cDNA was reverse transcripted by RTase (Invitrogen) and random N6 oligos, qPCR was performed using SYBR green PCR mixture from Roche, using primers of target genes or housekeeping gene β-actin.

For Northen blot analysis, total RNA (20 μg) was separated with the denaturing polyacrylamide gel, and transferred to N+-nylon membrane (Qiagen) by capillary method and cross-linked by ultraviolet treatment. After prehybridized with denatured DNA from salmon sperm, membranes were probed with the synthesized biotin labeled oligos of miR-147b or U6. Avidin-conjugated horseradish peroxidase was used to detect the hybridization signal.

### Analysis of cell proliferation

MTS and colony formation were used to detect cell proliferation. MTS assay were performed according to the user manual (Promega). For colony formation assay, cell was planted (200 cells/well) into 6-well plate in triplicate after transfection, and further cultured in for 10 days. After 15 mins fixing with methanol, colonies were stained with 0.1% crystal violet and quantitated by microscope counting.

### Luciferase reporter assay

After planting in 24-well plate for 18h, 293T cells were cotransfected with plasmids of luciferase reporter (200 ng) and Renilla luciferase (1 ng) together with the WT or mutated miR-147b. Cells were lysed 24 h after transfection and extracts were prepared for luciferase activity detection with the kit from Promega.

### Western blot

Tumor cell or tissue were lysed, sonicated and boiled at 95°C for 5 min in sample buffer and protein concentration was quantified. Proteins were separated by PAGE, then transferred to PVDF membrane and blocked with 5% nonfat milk. Western blot was performed with anti-UBE2N (sc-58452) and anti-GAPDH (sc-47778) antibodies and corresponding HRP conjugated secondary Ab (Promega).

### Nude mice subcutaneous xenograft studies

For subcutaneous xenograft model, Huh 7 or HepG2 cells (1^*^10^6^) were transfected with oligos of miR-147b or NC duplex, and then injected into the female nude mice from the back flanks subcutaneously, and tumor growth was examined over the course of 6 weeks. Mice were maintained in SPF conditions, at the end of experiment, the mice were anaesthetized with chloral hydrate (5%, 1.5ml/mouse) by intraperitoneal injection, and then euthanasia was performed by cervical dislocation. Experiments were performed according to the ethical guidelines for animal experiments and approved by the Institutional Animal Care and Use Committee of the Second Affiliated Hospital of Shenyang Medical College (Shenyang, China).

### Statistics

The results are presented as mean ± SEM (n=3). Unpaired t-test was applied for the statistical significance analysis between two groups; P value below 0.05 was considered significant.
